The article "Atomic resolution studies detect new biologic evidences on the Turin Shroud" was retracted in 2018. Reasons: a conflict of interest; bias or lack of balance; concerns about the data; concerns about the images.

# Atomic resolution studies detect new biologic evidences on the *Turin Shroud*

**DOI:** 10.1371/journal.pone.0180487

**Published:** 2017-06-30

**Authors:** Elvio Carlino, Liberato De Caro, Cinzia Giannini, Giulio Fanti

**Affiliations:** 1 Istituto Officina dei Materiali, Laboratorio Tecnologie Avanzate Superfici e Catalisi del Consiglio Nazionale delle Ricerche, Area Science Park–Basovizza, Trieste, Italy; 2 Istituto di Cristallografia, Consiglio Nazionale delle Ricerche, Bari, Italy; 3 Department of Industrial Engineering, Padua University, Padua, Italy; Institute of Materials Science, GERMANY

## Abstract

We performed reproducible atomic resolution Transmission Electron Microscopy and Wide Angle X-ray Scanning Microscopy experiments studying for the first time the nanoscale properties of a pristine fiber taken from the Turin Shroud. We found evidence of biologic nanoparticles of creatinine bounded with small nanoparticles of iron oxide. The kind, size and distribution of the iron oxide nanoparticles cannot be dye for painting but are ferrihydrate cores of ferritin. The consistent bound of ferritin iron to creatinine occurs in human organism in case of a severe polytrauma. Our results point out that at the nanoscale a scenario of violence is recorded in the funeral fabric and suggest an explanation for some contradictory results so far published.

## Introduction

The Turin Shroud [1] (TS) is a handmade 3–1 twill linen cloth, 4.4 m long and 1.1 m wide, showing the double image of a dead body of a scourged, thorn-crowned man who was stabbed in the side and crucified [2]. It is believed by many that it was the burial cloth in which Jesus of Nazareth was wrapped about 2000 years ago. Conversely, others think that it is a fake. However, the TS image has not been explained nor reproduced so far by science [3], although some hypotheses have been proposed [4]. There are some indications [5] that the TS was in Palestine in the first century A.D. and then taken to Edessa, now Sanliurfa (TR). The similarity of many details of the TS face with the Christ on Byzantine coins in use from the VII century A.D. is a clue that the TS were already known during the Byzantine Empire [3]. After the Sac of Constantinople in 1204 the “*Shroud of Christ*” appeared in Europe in 1353 at Lirey (F) [5] and in 1532 at Chambéry (F) where it was fire damaged [6]. It was taken to Turin in 1578 where it is still now.

In 1989 the linen fabric of the TS was radiocarbon dated to the Middle Ages [7]. This result is considered wrong by some authors claiming the presence of systematic errors [8]. Another work indicated an age for the TS “*between 1300-and 3000-years old*." [9] A mechanical analysis coupled with opto-chemical measurements has recently dated the TS to 90 AD ±200 years [10].

The article "Atomic resolution studies detect new biologic evidences on the Turin Shroud" was retracted in 2018. Reasons: a conflict of interest; bias or lack of balance; concerns about the data; concerns about the images.

The TS shows [1–3] a pale yellow background fabric, the body image—devoid of pigments [1,2,11]—produced by a chemical reaction (dehydration and oxidation) [1,2,11], blood stains and other localized signs of minor interest like burns, water stains etc. [1–3]. In 1969 Cardinal Pellegrino appointed a commission to investigate if the red stains clearly visible on the TS were blood. In 1973, a discordant conclusion was obtained: “*The negative response of the investigation does not allow an absolute judgment of exclusion of blood nature of the material*” [12]. Subsequent analyses of some TS threads evidenced only the presence of red pigments compatible with red ochre and vermillion, [13] whereas other researchers found the evidence of blood [14,15,16,17]. A recent study [17] found both blood and pigments proposing a retouch for the faded bloodstains. In summary, there is a strong controversial about the TS authenticity due to contradictory results of scientific analyses.

Up to now, to our knowledge, microscopic analyses on the TS were limited, at the best of times, to sub-micrometer spatial resolution.

Here we present an atomic resolution study on a fiber of the TS performed by Transmission Electron Microscopy (TEM) and Wide Angle X-ray Scanning (WAXS) Microscopy. The fiber, of about two millimeters, comes from an area of the feet (dorsal image) containing some red crusts, of about one micrometer, visible by optical microscope [17]. TEM experiments were performed in areas of the fiber away from red crusts.

TEM analyses show that the fiber is fully covered by creatinine nanoparticles, 20–100 nm in size, embedding small (2–6 nm) nanoparticles, made of defected ferrihydrite, typical of biologic ferritin cores. WAXS shows the presence of diffraction peaks of defected cellulose. Here we show how atomic resolution investigations unexpectedly discover a scenario of violence hidden at the nanoscale in the TS fiber and also suggest an explanation for the controversial results so far obtained. Indeed, a high level of creatinine and ferritin is related to patients suffering of strong polytrauma like torture. Hence, the presence of these biological nanoparticles found during our TEM experiments point a violent death for the man wrapped in the Turin shroud.

## Materials and methods

The fiber was provided by B. M. Schwortz [18], as part of the *Shroud of Turin Education and Research Association*, *Inc*. (STERA Inc). The fiber analyzed is taken from a sticky tape (1HB) applied to and lifted from the surface of the TS in 1978 [1]. We prepared the TEM specimen by placing the as received fiber, shown in Fig 1, in a folding 300x300 mesh Cu grid mounted on a further Cu grid previously covered by a thin C film “S1 Fig”. The measurements were performed in ultra-high vacuum of 7×10^−6^ Pa.

The article "Atomic resolution studies detect new biologic evidences on the Turin Shroud" was retracted in 2018. Reasons: a conflict of interest; bias or lack of balance; concerns about the data; concerns about the images.

**Fig 1:** Light microscopy image. Low-magnification, light microscopy dark-field, epi-illumination image of a piece of fiber of the TS: the arrows indicate some of the red particles on the surface of the fiber recognized as blood [17].

TEM experiments were performed at room temperature by using a JEOL JEM 2010F UHR TEM/STEM. The equipment has a low spherical aberration coefficient objective pole piece (Cs = 0.47±0.01mm) and has been operated at an accelerating voltage of 200 kV resulting in a spatial resolution of 0.19 nm at optimum defocus in phase contrast High-Resolution Transmission Electron Microscopy (HRTEM) imaging [19].

Energy Dispersive X-rays Spectroscopy (EDXS) experiments were performed in Scanning TEM (STEM) configuration by scanning an electron probe of 0.2 nm in the area of interest. The sample is extremely sensitive to the high-energy electron beam and has a high degree of hydro-carbon contamination [19] due to the prolonged exposure of the TS to the environment. These two conditions impose the use of a proper tailored electron-optical configuration capable to deliver a low current density onto the specimen [19,20]. The TEM experimental set up here used to study the TS fiber has been only recently established during the studies of pristine drug nano-crystals [21,22].

Wide Angle X-ray Scanning Microscopy (WAXS) data were collected at the X-ray MicroImaging Laboratory (XMI-L@b) equipped with a Fr-E+ SuperBright rotating anode copper anode microsource (Cu Kα, λ = 0.15405 nm, 2475 W), a multilayer focusing optics (Confocal Max-Flux; CMF 15–105) and a three-pinhole camera (Rigaku SMAX-3000) [23]. For WAXS data collection an image plate detector with 100μm pixel size was placed at 28mm from the sample and calibrated by means of the Si NIST standard reference material (SRM 640b) [24].

## Results

Fig 2 shows a High Angle Annular Dark Field (HAADF) STEM image in a false color output. This incoherent imaging approach enables to distinguish immediately regions of the sample with different average atomic number or thickness [25]. The small spots visible in Fig 2 are nanometric-sized particles covering the whole TS fiber (the arrows in the image point two areas where we prolonged the observation, producing circular large spots due to electron beam induced growth of carbon contamination [19]).

**Fig 2:** Low magnification High Angle Annular Dark Field STEM image. The smaller spots in the image are nanometric-sized particles surrounding the TS fiber. The arrows in the image point two areas of carbon contamination due to prolonged exposure to the electron probe.

The article "Atomic resolution studies detect new biologic evidences on the Turin Shroud" was retracted in 2018. Reasons: a conflict of interest; bias or lack of balance; concerns about the data; concerns about the images.

Extended TEM/STEM experiments make evident that the TS fiber is widely covered by nanoparticles with sizes between 30nm to 100nm. These nanoparticles contain inside small structures, with size ranging between 2nm and 6nm, characterized by a dark contrast in the HRTEM images, as shown in a representative result in Fig 3 (see also for further examples S2 Fig). In particular, in Fig 3 it can be distinguished the large nanoparticle, in this case about 90 nm in size, with a lighter contrast with respect to the small dark particles inside it, which are 2–6 nm in size.

**Fig 3:** Representative HRTEM image for nanoparticles covering the fiber. Representative HRTEM image in a false color output of one of the big nanoparticles covering the TS fiber. Note the small dark particles, with diameters between 2nm and 6nm, inside.

In Fig 4 it is reported a Wide Angle x-ray microdiffraction pattern (green profile) collected within a total scanned area of 1.22x1.22 mm^2^. The experimental WAXS profile was compared with the convolution (black curve) of the theoretical diffraction patterns of two cellulose structures (COD #4114994 and COD # 4114382), which have similar lattice spacing. The large full width at half maximum of the experimental main (002) peak can be related to the amount of defects present in the cellulose structure [26], as expected for the age of the TS fiber. The additional experimental profile corresponds to cellulose fibers of the VI century (blue profile), sample D in reference [10], which have been measured to verify the effect of the aging on the peak visibility.

**Fig 4:** WAXS pattern. Azimuthally integrated experimental WAXS pattern (green curve) compared to the cellulose theoretical diffraction pattern (black curve). For comparison, cellulose WAXS pattern was collected also on fibers of the VI century (blue profile), sample D in reference [10].

The atomic resolution HRTEM experiments at the nanoscale enable to access a range of TS features never explored so far. The morphology and the size of the particles detected on the TS fiber, see Fig 3 and S2 Fig, are very similar to those of proteins like hemosiderin [27], or to ferritin-based proteins typical of blood [28,29,30].

EDXS experiments performed on individual large particles, as the one shown in Fig 3, reveal the presence of Ca, O, C, N, Fe, S, K, Cl (see S3 Fig), which are compatible with ferritin-based proteins [31,32]. Nevertheless, the high contamination rate [19] due to the century exposure of the TS to the environment does not permit to have enough statistics to discriminate and quantify the EDXS signal coming from the small dark particles with respect to those coming from the big particles embedding them. Therefore, to identify the nature of each nanoparticle we analyzed the atomic resolution HRTEM images and the diffractograms of individual particles [21,22].

The article "Atomic resolution studies detect new biologic evidences on the Turin Shroud" was retracted in 2018. Reasons: a conflict of interest; bias or lack of balance; concerns about the data; concerns about the images.

HRTEM experiments revealed the crystalline nature of all kinds of nanoparticles. The HRTEM analysis, when focused on individual small dark particles lead to measure lattice spacing of 0.37 nm, 0.36 nm, 0.35 nm, 0.31 nm, 0.30 nm, 0.23 nm, 0.22 nm, 0.21 nm, 0.17 nm. The measurements are affected by an experimental uncertainty less than 3%. These spacing are compatible with those of some iron oxides [28]. Many of the diffractograms exhibit more than one Friedel’s pairs, related to entangled crystalline symmetries and spacing, representing the signature of the analyzed structures [21,22] and enabling an accurate structure identification and simulation.

Fig 5 shows a representative HRTEM image focused on a small dark nanoparticle (panel a), zoomed in panel b, together with its corresponding high symmetry diffractogram (panel c) and relevant simulation (panel d). The reciprocal space pattern in Fig 5C has symmetry and spacing in agreement with the [4 2 1] zone axis of six-line ferrihydrate (a = b = 0.59nm; c = 0.91nm; α = β = 90°; γ = 120°; P63mc space group) [33] as evident in comparison with the simulation in panel d). It is worthwhile to remark that the six-line ferrihydrite iron oxide has been proposed for the core of the iron-storage ferritin [34,35]. Other examples and crystal orientations are shown in S4 Fig.

**Fig 5:** Representative results on the small dark particles. a) HRTEM image focused on one of the small and dark nanoparticles shown in Fig 3; b) zoom inside the red square of panel a) (false color output); c) diffractogram relevant to the zoomed area in panel b); d) simulation, with the Miller indexes associated to some spots and the corresponding lattice spacing. Simulations show that the diffractogram of panel c) is compatible with the ferrihydrate in the [4 2 1] zone axis.

The peculiar structure, size and distribution of the iron oxide nanoparticles that we found on the TS fiber are very important in the debate about the presence of artifacts on the relic, since they enable to exclude ancient dye for painting. Indeed, ancient dye pigments are, in general, on the scale of hundreds of nm [36]. Even if painting dyes of few nanometers had been used, they would be not well dispersed inside big nanoparticles, as observed in our experiments (see Fig 3 and S2 Fig), but they would tend to aggregate each other [37]. This is an important experimental evidence here achieved thanks to the high spatial resolution of TEM, since so far only *sub-micron particles* were observed in the TS [13,17]. The particles observed in some previous works evidenced the human intervention with red ochre and vermillion used over bloodstains, but organic and inorganic particles have sizes [13,17] at least one hundred times bigger than those observed in our HRTEM studies.

The article "Atomic resolution studies detect new biologic evidences on the Turin Shroud" was retracted in 2018. Reasons: a conflict of interest; bias or lack of balance; concerns about the data; concerns about the images.

## Discussions

There is a strange occurrence that we noted during all of our TEM studies. In fact, although HRTEM experiments evidenced how the dark small nanoparticles are made of ferrihydrite, nevertheless in all of our TEM experiments, the peculiar spacing of iron oxide at 0.25 nm [28] was oddly never observed. The absence of the 0.25nm spacing could be due to the interaction between the small iron-oxide particles and the particle embedding them, which from one side prevented their modification during the centuries due to the interaction with the external environment, but could have affected some of the peculiar crystal features of the iron oxide clusters.

Indeed, the explanation comes from some recent studies on the binding between creatinine and urea with iron-oxide nanoparticles investigated, in a completely different field, for possible application in dialysis to reduce waste molecules accumulation in blood [38]. In particular X-ray studies on iron oxide nanoparticles tagged with urea and creatinine indicate exactly a suppression of the Bragg diffraction peak corresponding to the 0.25nm spacing [38]. We hence focused our attention to identify the structure of the big embedding nanoparticles comparing their HRTEM images and diffractograms with the relevant full dynamical calculations of diffraction patterns for urea and creatinine [39]. As a result, all the identified diffractograms belong to creatinine. A representative example of our findings is shown in Fig 6 (see also S5 Fig for other examples).

**Fig 6:** **Characterization of creatinine particles** a): HRTEM image; b): magnified view of the square region marked in a); c): diffractogram of b); d): simulation of the diffraction pattern of creatinine in [1–10] zone axis with reported the lattice spacing relevant to the observed intensities. The yellow and pale-blue circles in the diffraction pattern simulation mark the corresponding circles around the experimental spots in c).

We measured the diffractogram (Fig 6, panel c) in the area marked by a square in the relevant HRTEM image (panel a) and shown at higher magnification in panel b). In the TEM experiments we focused the attention on those particles oriented with respect to the electron beam to excite more than one pair of reflections. This enables to unambiguously identify the relevant zone axis and material structure [40,21,22]. The diffractogram in Fig 6 belongs to creatinine oriented along the [1–10] crystallographic zone axis with respect to the direction of the direct electron beam, as demonstrated by the relevant diffraction pattern simulation shown in Fig 6D. In the latter, for ease of reading, we highlighted those reflections that enable the identification of the creatinine removing the systematic reflections that are not transmitted, or poorly transmitted, by the contrast transfer function of the objective lens [19,20]. The yellow and pale-blue circles in the diffraction pattern simulation mark the corresponding circles around the experimental spots in Fig 6C. The yellow circles and the pale-blue circles in the diffractogram point two independent pairs of reflections, whose spacing is respectively of 0.59nm and 0.23nm, forming a reciprocal space angle of 94 degrees. These two Friedel’s pair correspond respectively to (002) and (22–1) spots of creatinine, as shown in the relevant simulation. Other examples, also in other particle crystallographic orientations, are given in S5 Fig. Hence, on the basis of the experimental evidences, the particles covering the TS fiber are creatinine nanoparticles with inside biological ferritin cores of ferrihydrate. The lack of the 0.25nm spacing evidenced during our experiments is due to the bond between ferrihydrate cores and creatinine in agreement with the evidences in the x-ray spectra of the creatinine bounded to iron oxide nanoparticles where the peak corresponding to the spacing at 0.25nm is suppressed by the interaction between the protein and the iron [38].

The article "Atomic resolution studies detect new biologic evidences on the Turin Shroud" was retracted in 2018. Reasons: a conflict of interest; bias or lack of balance; concerns about the data; concerns about the images.

This is not a situation typical of the blood serum of a healthy human organism. High levels of creatinine in the blood are observed in the case of strong trauma. There is a wide recent literature reporting on interaction between creatinine and ferritin in fatal accidents [41,42] or as a consequence of the rhabdomyolysis due to torture [43]. Indeed, De Abreu et al. report in [41] a study on acute kidney injury (AKI) after trauma, mostly in accidents involving cars and motorcycles, evidencing how AKI is secondary to severe crush injuries and rhabdomyolysis. In particular, the patients with AKI present a high level of creatinine and ferritin in the blood serum. High level of creatinine are also in the case reported by Schwartz et al [42] in the study of patients of emergency room with skeletal muscle trauma. Indeed, when muscle cells are destroyed as a consequence of a strong trauma, such as the torture, they release their content into the bloodstream as reported in [43]. One of the chemicals largely released is myoglobin [43]. The creatinine strongly binds to the iron nanoparticles [38] of the ferritin and this relationship is hence a signature of the occurrence of a strong polytrauma.

The article "Atomic resolution studies detect new biologic evidences on the Turin Shroud" was retracted in 2018. Reasons: a conflict of interest; bias or lack of balance; concerns about the data; concerns about the images.

## Conclusions

On the basis of the experimental evidences of our atomic resolution TEM studies, the man wrapped in the TS suffered a strong polytrauma. We studied a fiber of the TS by atomic resolution TEM experiments and WAXS. This is the first time that the TS is studied at this resolution and this range of view produced a series of experimental results, which thanks to recent studies on ancient dye painting, ferritin, creatinine and human pathology can be connected and understood in relationship with a macroscopic scenario in which the TS was committed [41,42,43]. In fact, the fiber was soaked with a blood serum typical of a human organism that suffered a strong trauma, as HRTEM evidenced that the TS is covered by well-dispersed 30nm-100nm creatinine nanoparticles bounded with internal 2nm-6nm ferrihydrate structures. The bond between the iron cores of ferritin and creatinine on large scale occurs in a body after a strong polytrauma [41,42,43]. This result cannot be impressed on the TS by using ancient dye pigments, as they have bigger sizes and tend to aggregate, and it is highly unlikely that the eventual ancient artist would have painted a fake by using the hematic serum of someone after a heavy polytrauma. Nevertheless, the presence of red pigments, detected in some studies [13,17] seems to indicate a human intervention on the TS. This, in turn, has generated some difficulties for the modern investigations and stimulated the scientific debate about the actual origin of the TS. The analyses discussed in literature so far, have been realized without the necessary spatial resolution to distinguish what is coming from the nanoscale and cannot filter eventual artifacts. This has been the target of our work and the obtained results are not compatible with a painting but evidenced the presence of nanoparticles of pathologic blood serum related to the presence of creatinine bound with ferrihydrate, which are typical of an organism that suffered a strong polytrauma, like torture. Indeed, unexpectedly, at the nanoscale it is encoded a scenario of great suffering recorded on the nanoparticles attached to the linen fibers. Furthermore, here the experiments point how the nanoscale enable to study unspoiled properties of the Turin Shroud suggesting an effective experimental strategy for further studies.

## Supporting information

S1 Fig TEM image. Low magnification TEM image of part of the TS fiber, pointed by blue arrows, surrounded by the bars of the TEM Cu grids marked by red straight lines. For reader convenience we place in the inset a light optical image of a TEM grid with diameter of 3mm.
(TIFF)

S2 Fig HRTEM images. Low Magnification HRTEM image of further examples of big particles, containing iron oxide small dark clusters.
(TIFF)

S3 Fig EDXS spectrum. Representative EDXS spectrum as acquired on individual large particle of the kind shown in Figs 3 and S2.
(TIFF)

S4 Fig Experimental diffractograms. Further examples of high symmetry diffractograms, with different crystal orientations, belonging to ferrihydrate small particles.
(TIFF)

S5 Fig Experimental diffractograms. Further examples of diffractograms of creatinine.
(TIFF)
